The article "Improvement of the Public Health Service Platform System Based on the Big Data-Driven System" was published in 2022. Journal: Comput Intell Neurosci.

# Improvement of the Public Health Service Platform System Based on the Big Data-Driven System

**DOI:** 10.1155/2022/1476779

**Published:** 2022-07-06

**Authors:** Hua Tian

**Affiliations:** School of Intelligence & Electronic Engineering, Dalian Neusoft University of Information, Dalian, Liaoning 116023, China

## Abstract

At present, complex discrete dynamic systems are widely used in the field of medicine. The control system in the complex discrete dynamic model is gradually transformed into intelligent control. It has become the main research direction of researchers to improve the medical platform system by adding different modeling strategies. The traditional discrete modeling technology can only be used as the knowledge content of students' textbooks because it can no longer meet the needs of the development of human society. In order to improve the application of a discrete system in the public platform, this paper studies the improvement of the public health service platform system based on the complex discrete dynamic system. Firstly, a time-driven control strategy is proposed to study the output feedback control with random sampling in the platform. Then, the stability of random parameters and the addition of dynamic scheduling strategies are further studied. Compared with the traditional system, the optimized system greatly strengthens the data transmission problem of input and output channels. The results show that by improving the performance of the public health service platform system, the probability of problems in the process of data transmission is greatly reduced. After adding controllable and observable performance to the system, the stability of the whole system is further improved. The improved public health service platform system studied in this paper can store and transmit a large number of user data in the network environment, automatically maintaining the stability of the system and has a good social application value.

## 1. Introduction

With the progress of today's era, the performance of complex discrete dynamic systems has been continuously improved [1]. In different application fields, the methods of system improvement are also flexible. The complex discrete dynamic model with different improved technologies is widely used in the transportation industry, the aerospace industry, the medical service industry, and other fields [2]. In the field of the medical industry, because the population is huge, a large data system is required. Therefore, complex discrete dynamic modeling technology is widely used in the medical service platform system [3, 4]. When the modeling technology was first applied, many researchers only added the basic technology of input and output data. However, when dealing with data, this common complex discrete dynamic modeling technology often has many problems, such as system error, collapse, data information, and confusion [5]. Once the above problems occur, the system of the whole service platform can no longer be used. In order to solve the above problems, researchers subsequently proposed optimization technology to improve the optimization data processing ability in discrete dynamic systems. The improvement of this ability does make the system less prone to system crash and data confusion in the state of processing data [6]. However, the use of this optimization technology has become particularly picky about the user's data requirements, which also brings great trouble to the user in the process of use. Later, many researchers solved various data problems of the system by adding output feedback control technology and data stabilization technology. Subsequently, by adding dynamic scheduling strategy, the whole platform system can always maintain a stable operation environment for processing data [7]. Through the combination of three optimization technologies and models, the whole service platform system also improves the efficiency. Secondly, the platform system can also effectively process the data entered by users [8].

In recent years, with the rapid development of optimization complex discrete dynamic modeling technology, optimization technology has evolved into various forms in all walks of life [9]. In recent years, researchers have applied the output feedback control technology of the optimization system to different kinds of data systems [10]. In the optimized complex discrete dynamic system, it can comprehensively process the output data so as to improve the work efficiency of the whole model system. On the premise of the above contents, based on the complex discrete dynamic modeling technology, this paper puts forward the output feedback control technology and the stability technology of the system and data [11]. The above technologies can improve the system performance of the public health service platform studied in this paper [12]. The upgraded platform system can maintain normal system operation under the processing of massive data and various environmental factors, greatly reducing the maintenance cost of the system [13].

This paper studies the improvement of the public health service platform system based on the complex discrete dynamic system. The innovation contribution includes research and puts forward the improvement scheme of the public health service platform. By strengthening the stable state between the system and data, errors and failures are reduced. By adding the output feedback control scheme, the error reduction strategy is adopted to improve the accuracy of the data. Adding the public health service platform under the output feedback control scheme can greatly reduce the error in the data processing process. Through the analysis of public system stability and system transmission stability, the combined public health service platform has significantly improved the data processing speed and system stability.

This paper is mainly divided into three parts. The first part is a brief description of the related technology and development of optimizing complex discrete dynamic systems. The second part is the performance optimization of complex discrete dynamic modeling based on the health service platform. Firstly, the output feedback control problem of the network control system is studied. Based on the discrete dynamic model driven by the Markov chain, the controller and transmission strategy are added to the input and output of data for optimization. Finally, it is proposed to stabilize the system and optimize the stability of the scheduling transmission of the system. The third part analyzes the research results of output feedback control optimization in the health service platform system, as well as the optimization results of data stabilization and system scheduling and transmission performance.

## 2. The Related Works

The public health service platform system is based on complex discrete dynamic modeling technology. Firstly, the medical information data input by the user is analyzed and stored, and finally, the data input by the user is output to achieve the purpose of system use [14]. In the data input by users, it is necessary to systematically process the data. The information of each user is different, and the output data will be unstable in the process of data analysis and processing [15, 16]. In order to avoid the problem of output mismatch when each user uses the system, researchers have proposed a complex discrete dynamic model with a controller in recent years [17]. The main core content of controller technology is to maintain the state stability of the input and output data and the whole service platform system. However, by adding the controller, the whole discrete dynamic system and data cannot reach a completely stable state. Later, many researchers also introduced the observer and dynamic scheduling strategy on the basis of the controller and obtained a more stable system state [18]. Through the addition of the above optimization technology, the platform system under the complex discrete dynamic model can better process the data information, reduce various internal and external factors affecting the data, and finally realize the optimal construction of the service platform [19].

Complex discrete dynamic technology is widely used in the aerospace field. As we all know, the United States is a big country with economic development and is the first country to achieve success in the field of manned aerospace [20]. Astronauts collect samples on the moon and send all kinds of data obtained from sample research to the base. The received data are deeply analyzed and processed through complex discrete dynamic systems, which provide good help to relevant researchers.

Complex discrete dynamic systems are usually used in the production and product monitoring of skin care products. The safety of skin care products and food safety are equally important to human beings, through the monitoring of added components and usage in skin care products [21]. Once the dosage of an additive exceeds the standard, the production monitor will find the product problem from the data in the computer for the first time. The reference of the system is also a major breakthrough in product safety.

Complex discrete dynamic systems are also mainly used in the field of water quality detection [22, 23]. As China's population ranks first in the world, the drinking water problem of Chinese people has always been a big problem to be solved. In the water quality detection of new water sources, through the introduction of this technology, the water quality data can be automatically compared with the original data, thus greatly reducing the labor force. The data information such as money, date, and account accessed by many users can be classified [24]. Moreover, it can also let customers know their account information in real time by combining it with the Internet. The introduction of this technology is conducive to promoting the development of economy and industry. According to the application of complex discrete systems in the above countries, this paper studies the improvement of the public health service platform system based on complex discrete modeling technology. Finally, the system performance of the public health service platform is optimized [25]. In the optimization process, the data output control function is added to the system, and then, the data observer is added. Finally, the networked system stability technology is used to optimize and improve the public health service platform.

## 3. Research on Improvement of the Public Health Service Platform System Based on the Big Data-Driven System

### 3.1. Analysis on Output Feedback Control of the Public Health Service Platform System

Markov chain driving reduces the conservatism of the system when processing data. The main reason is that the optimal design of data output feedback control in the system is mainly driven by the Markov chain. The design can perform stable data output operation on the data input to the system and ensure that the core content of the output feedback control structure is to maintain the stable state of the closed-loop system [26]. The stability of the networked system is maintained by adopting the drive transmission strategy at the data input and the design of the time-delay bidirectional system controller. The traditional process optimization technology of the data processing algorithm mostly uses the small double algorithm [27]. The algorithm mainly optimizes the processing of sample data and can still maintain the normal data processing capacity on the basis of massive data. However, when the algorithm is applied to the software system under the discrete dynamic model, the data processing ability of the system is not very ideal, and the output results are very different every time [28]. It is also confirmed that the algorithm is affected by background environmental factors and cannot ensure the stability between the output data and the system. Based on the above situation, this paper proposes to optimize the user data output feedback control in the system. The structure of output feedback control is shown in Figure 1.

It can be seen from Figure 1 that the random sampling model is used in the structure of output feedback control, which can better observe the data randomness of the communication network. Data sampling is usually caused by the change in the load in the communication network. When the network in the system enters the working state, the data collector cannot continue to collect data information with high frequency, resulting in the extension of the working time of the system. In order to avoid the above problems, a nonslot technology is added. The algorithm flowchart is shown in Figure 2.

As can be seen from Figure 2, the algorithm combines the random data sampling model and the normal data sampling model. The data are processed through the algorithm. When the system is busy, it enters the random data sampling model, and when it is not busy, it directly outputs the data. By reducing network channel resources and communication times, the work efficiency of the service platform system is increased. In order to further improve the transmission rate of the wireless channel, the error reduction strategy and the optimization means of the controller are used [29]. The relevant formula is as follows:

(1) $$\begin{array}{c} L\left(\tau_{k-1},\tau_{k}\right)\left(y\left(k-\tau_{k}\right)-\overset{\wedge }{y}\left(k\right)\right),\\ \overset{\wedge }{x}=Ax\left(k\right)+Bu\left(k\right)+L\left(\tau_{k-1},\tau_{\text{k}}\right)-y\left(k\right),\\ \overset{\wedge }{y}=Cx\left(k\right),\\ u\left(k\right)=Kx\left(\tau_{k-1},\tau_{k}\right),\\ x\left(0\right)=0. \end{array}$$

Through the above formula, the error between the platform system and the observer is reduced, and the output controller is established, which can predict the state of the system more accurately. The software simulation model of the controlled object is used as the executing control loop, and the output signal of the power converter acts on the actual controlled object and the estimation model of the controlled object at the same time. The optimization technology is added to the controller and the observer in the output channel. The formula of the extended dimension platform system is as follows:

(2) $$\begin{array}{c} \left\{\begin{array}{c} X\left(k+1\right)=\bar{A}X\left(k\right)+\bar{B}u\left(k\right),\\ X\left(k+1\right)=\bar{A}X\left(k\right)+\bar{B}u\left(k\right)+L\left(\tau_{k-1},\tau_{k}\right)\left(CR\left(\tau_{k}\right)X\left(k\right)-Cx\left(k\right)\right). \end{array}\right. \end{array}$$

Combined with the extended dimension platform system formula, the closed-loop system formula is derived:

(3) $$\begin{array}{c} Z\left(k+1\right)=\left(\overset{\wedge }{A}+\overset{\wedge }{B}G_{\left(K,L\right)}\left(\tau_{k-1},\tau_{k}\right)\overset{\wedge }{C}\left(\tau_{k-1},\tau_{k}\right)\right)Z\left(k\right). \end{array}$$

Based on the above technical support, the optimized complex discrete dynamic system is applied to the public health service platform, and the construction model of the public health service platform is obtained, as shown in Figure 3.

As can be seen from Figure 3, the construction model of the public health service platform transmits the user's information and service content through the Internet. This makes it possible for medical services to cross regions and systems. However, there will be various uncontrollable environmental factors in the network-based service system [30]. In this paper, the platform system controller is added to the whole platform system to further control the system disorder caused by environmental factors. The controller needs to satisfy relevant inequalities, and the formula is as follows:

(4) $$\begin{array}{c} \left[\begin{array}{ccc} -p\left(i\right) & {\left(i,0\right)}^{T} & {\left(i,i+1\right)}^{T}\\ {}* & -ϒ\left(0\right) & 0\\ {}* & * & -ϒ\left(i+1\right) \end{array}\right]<0,\\ \left[\begin{array}{ccc} -p\left(i\right) & {\left(i,0\right)}^{T} & {\left(i,i+1\right)}^{T}\\ {}* & -ϒ\left(0\right) & 0\\ {}* & * & -ϒ\left(i+1\right) \end{array}\right]<0, \end{array}$$

ϒ in the inequality must satisfy the following conditional formula:

(5) $$\begin{array}{c} ϒ\left(N\right)={\left(\pi_{N0}P\left(N\right)\right)}^{-1}. \end{array}$$

Based on the construction method of the system controller and nonlinearity between controllers, the following formula is obtained:

(6) $$\begin{array}{c} \left[\begin{array}{cc} P\left(i\right) & I\\ {}* & ϒ\left(i\right) \end{array}\right]\geq 0,\;i\in \left\{0,1,2,\ldots ,N\right\}. \end{array}$$

According to the iterative algorithm and the above formula, the data information in the system is calculated. The final data result is the required data gain between system controllers. After adding the output control optimization scheme to the platform system, the system performance is experimentally explored based on the packet loss of processing data. The exploration results are shown in Figure 4.

It can be seen from Figure 4 that when the optimized service platform system is in the working state, the stability of the user data and complex discrete dynamic model in the platform system can be seen from the relative ratio of the data packet loss in the output channel to the normal packet loss. To sum up, by adding an output feedback controller to the public health service platform system, the system can carry out stable and efficient circular operation from the information data generated by service users.

### 3.2. Optimization of Stabilization and Scheduling Transmission Stability of the Public Health Service Platform System Based on the Big Data-Driven System

In the public health service platform driven by big data, system stabilization and scheduling transmission stability optimization are also important. In complex discrete dynamic systems, because the Markov packet loss will occur at the output, variable objects are introduced to describe the packet loss of the Markov user data when data information is output. By adding a multidensity quantizer and increasing the width of the measured values, the stability condition of the closed-loop system is finally achieved. In the networked system, the observer measures the data in the discrete dynamic system, constructs the random parameters through the measured values, and finally introduces the parameters into the transmission model. In the service platform system studied in this paper, each channel is independent of each other, and the error of the measurement results can be quantified in the data packet loss measurement. Firstly, the model formula and random parameters of the complex discrete system are set as follows:

(7) $$\begin{array}{c} x\left(k+1\right)=A\left(k\right)x\left(k\right)+Bu\left(k\right),\\ A\left(\alpha \left(k\right)\right)=A+\bar{A}\left(k\right). \end{array}$$

After calculating the random data parameter value in the complex discrete system, in order to further describe the data packet loss value, the transmission model of the complex discrete system and the related algorithms to describe the packet loss are added. The following formula is

(8) $$\begin{array}{c} \bar{y_{i}}\left(k\right)=\theta_{i}\left(k\right)y_{i}\left(k\right),\;i\in \psi^{a},\\ \delta \left(k\right)=\sum_{i=1}^{s}\theta_{i}\left(k\right). \end{array}$$

It is considered that the measurement error will occur when the system measures the parameter value of the data packet loss. If the error is not quantified, the final outgoing packet loss data are also inaccurate, which will affect the wrong judgment of the system performance of the service platform. The relevant formulas for error quantization processing are as follows:

(9) $$\begin{array}{c} \varsigma_{ij}\left(k\right)=q_{ij}\left(v_{i}\left(k\right)\right)-v_{i}\left(k\right). \end{array}$$

After measuring the data packet loss through the above formula, the data are transmitted to the computer, the data are systematically calculated in the input channel, and finally, the input channel capacity suitable for the system is obtained. In this experiment, the average channel capacity and real channel capacity are systematically calculated, respectively, as shown in Figure 5.

It can be seen from Figure 5 that the difference between the average channel capacity and the real channel capacity does not exceed 0.2. It can be seen from the value of the phase difference that the real data channel capacity is very close to the average channel capacity. The data channel with large capacity will improve the data transmission efficiency. In order to be able to transmit in the wireless network, we can still analyze and detect the performance stability of the public health service platform system studied in this paper, mainly through the breadth increase in the Markov packet loss value, and the breadth increase equation is as follows:

(10) $$\begin{array}{c} \delta \left(k\right)=\sum_{i=1}^{s}\theta_{i}\left(k\right)\\ =\sum_{i=1}^{s}\bar{\theta_{i}}\left(r\left(k\right)\right)\\ =\bar{\delta }\left(r\left(k\right)\right). \end{array}$$

The addition of this equation reduces the complexity of subsequent verification and optimization of platform system performance. After optimizing the performance of the Markov packet loss value, this paper explores the trajectory of the Markov packet loss value between the system and the observer as shown in Figure 6.

It can be seen from Figure 6 that the optimized Markov data packet loss value is very stable in the platform system. It can be seen from the system data observer that the Markov data packet loss value fluctuates all the time, but the fluctuation peaks correspond to it. Generally speaking, the Markov data packet loss value remains in a stable state.

Because the number of users faced by the public health service platform studied in this paper is immeasurable, the capacity of the channel is optimized. When the service platform is in the system communication constraint environment, in order to solve the behavior of data constraints, this paper adopts the dynamic communication scheduling method. The dynamic communication scheduling method formula is as follows:

(11) $$\begin{array}{c} y_{1}\left(1\right),y_{2}\left(2\right),\ldots y_{q}\left(n_{1}\right),y_{2}\left(n_{1}+1\right),y_{2}\left(n_{1}+2\right)\ldots ,\\ y_{2}\left(n_{1}+n_{2}\right),\ldots ,y_{q}\left(n_{1}+\cdots +n_{q-1}+1\right),\\ y_{q}\left(n_{1}+\cdots +n_{q-1}+2\right),\ldots . \end{array}$$

Disadvantages of static routing are as follows: in a complex network environment, the number of operations is very large. It has low adaptability to the complex network environment. Advantages of dynamic routing are as follows: small maintenance and strong adaptability. The reason why this paper does not use the static communication transmission method is that the static scheduling method cannot meet the controllability and observability of the platform system. Therefore, by using the dynamic communication transmission method, this method effectively solves the related problems of limited data in the communication process. By adding the dynamic scheduling method to the platform system, the capacity of the whole channel also changes. With the change in the channel capacity, the system stability region also changes as shown in Figure 7.

As can be seen from Figure 7, the stability of the optimized platform system has been greatly improved. After adding the dynamic scheduling method, the channel capacity of the system also increases by nearly one-third of the area. The system can also serve more users in a limited time, which strengthens the efficiency of the system.

## 4. Analysis of Research Results on System Improvement of the Public Health Service Platform Based on the Big Data-Driven System

### 4.1. Analysis of Research Results on System Output Feedback Control Optimization of the Public Health Service Platform Based on the Big Data-Driven System

Based on the optimized public health service platform system under the big data-driven system, this paper selects the data information of 2000 users in a hospital database as the experimental sample data. By inputting the sample data into the system with output feedback control and the ordinary control system, the performance of data processing is compared. The sample data are also put into the double-optimized service platform system X1, the optimized data processing service platform system X2, and the ordinary data processing system X3, and the performance test experiments are carried out, respectively. In the optimized system, firstly, the error reduction strategy is used to effectively control the output data to ensure that the error generated by the data is within the controllable range. Then, the output feedback controller is added to the system to ensure that the output data will not be affected by external uncontrollable environmental factors. Finally, through the combination of the two technologies, the goal of data optimization processing of the public health service platform is completed. In the experiment, the error of the output data and the efficiency of data processing are analyzed. The data processing comparison of different output feedback control systems is shown in Figure 8. The data errors in the three system states are shown in Figure 9.

As can be seen from Figure 8, the system with output feedback control is very efficient in processing sample data. The system without output feedback control is prone to data congestion, and the efficiency of data processing decreases obviously. In contrast, the system with output feedback control is more suitable for the subject studied in this paper. As can be seen from Figure 9, among the errors generated under three different system states, the error generated by the double-optimized service platform system X1 is the smallest and closest to the equilibrium state. The service platform system X2 for optimizing data processing does not include relevant technologies to stabilize the system. The error amount fluctuates greatly, but it is better than the ordinary data processing system X3. To sum up, the performance of the double-optimized service platform system is very suitable for this paper.

### 4.2. Analysis of Research Results on Stabilization and Scheduling Transmission Stability Optimization of the Public Health Service Platform System Based on the Big Data-Driven System

In the process of internal enhancement of the stabilization and transmission stability of the public health service platform system, this paper studies the scheme by measuring the packet loss value and dynamic transmission. Because the sample data processing efficiency of different platform systems is different, it is necessary to further verify the working efficiency of the public health service platform and increase the stability and transmission stability. Therefore, five groups of sample data with different capacities are prepared in this experiment. The five groups of data are mainly used for data input and output processing in the ordinary platform system, the platform system with scheduling transmission stability, and the platform system with stabilization performance and transmission stability performance. In the process of data processing, the system first measures the packet loss data, and the measured value is returned to the system through system mapping. Secondly, the system quantifies the error of the measured value of the packet loss data. Finally, the system dynamically transmits the normal data and outputs the results. The performance changes in three different systems in processing user data are shown in Figure 10.

It can be seen from Figure 10 that the platform system with stabilization performance and transmission stability can still carry out high performance and stable work efficiency when processing large-scale data. The processed user data can also ensure clarity and accuracy. Therefore, this paper proposes to add stabilization performance and transmission stability performance to the public health service platform for system improvement.

## 5. Conclusion

Nowadays, complex discrete dynamic systems are widely used in many fields, such as aerospace, public transportation, education, and artificial intelligence. The complex discrete dynamic systems can also optimize and upgrade the system according to different performance requirements. With the emergence of complex discrete dynamic modeling technology, the traditional discrete modeling technology can only be used as the knowledge content of students' books because it can no longer meet the needs of the development of human society. For example, when analyzing data, it may have a serious impact on the final output result due to the change in the data scale and state. Based on the above development, this paper proposes to improve the public health service platform based on complex discrete dynamic modeling technology. By strengthening the stable state between the system and data, the occurrence of errors and faults is reduced. Firstly, by adding the output feedback control scheme, the error reduction strategy is adopted to improve the accuracy of the data. The results show that adding the public health service platform under the output feedback control scheme can greatly reduce the error in the process of data processing. Finally, two performances are added based on the above scheme, namely, system stabilization and system transmission stability. The experimental results show that the combined public health service platform has significantly improved in the data processing speed and system stability. The research has a certain development and reference value, but there are still some limitations. The existence of recoverable faults increases the complexity of the system. In this paper, the discrete event dynamic system including time series and self-recoverable faults is not analyzed, so it needs to be further modified in the future research.

## Figures and Tables

**Figure 1:** Output feedback control structure diagram.

**Figure 2:** The flowchart of the nonslot algorithm.

**Figure 3:** Medical service platform.

**Figure 4:** Comparison diagram of the system packet loss diagram.

**Figure 5:** Input channel capacity diagram.

**Figure 6:** Trajectory of the system and observer x1.

**Figure 7:** The stability region of the closed-loop system.

**Figure 8:** The comparison diagram of the output feedback control processing data.

**Figure 9:** Data error of three system states.

**Figure 10:** The performance diagram of the optimized three different systems for processing user data.

## Data Availability

The data used to support the findings of this study are available from the corresponding author upon request.
